# Accidental Stainless Crown Ingestion During Dental Treatment in a Pediatric Patient

**DOI:** 10.7759/cureus.21335

**Published:** 2022-01-17

**Authors:** Yazeed M Almuaytiq, Ghazi L Alharbi, Sami A Alfahad, Sreekanth K Mallineni

**Affiliations:** 1 College of Dentistry, Majmaah University, Almajmaah, SAU

**Keywords:** crown, pediatric preventive dentistry, children, stainless steel crowns, ingestion

## Abstract

Accidental ingestion of foreign bodies is very frequent in children. Ingestion of dislodged restorations, dental appliances, crowns, and teeth in dental operatory is frequently reported. Early diagnosis of foreign bodies ingestion in a dental operatory and awareness of its signs and symptoms are very crucial. A five-year-old boy accidentally ingested a stainless steel crown during the trial fit at the dental operatory. Crown retrieval was attempted but without success, and thus, the patient was further observed for possible signs and symptoms. Due to possible serious complications, ingestion of foreign bodies during dental procedures must be appropriately prevented and managed if it occurs.

## Introduction

Accidental ingestion of foreign bodies is one of the most common problems in young children [1]. This accidental ingestion poses them at a higher risk of aspirating or swallowing various household objects [2]. In the dental operatory, accidental ingestion occurs in geriatric and pediatric patients and has been very commonly reported in children [3]. Ingestion of materials and appliances in dental operatory sometimes may end up with serious complications. Clinical signs and symptoms of such children are to be monitored meticulously until the foreign body passes through the gastrointestinal tract (GIT) [4]. It might sometimes become necessary to intervene with a surgical procedure. Tamura and co-workers reported that the frequency of dental-related objects ingestion ranges from 3.6% to 27.7% among all foreign bodies [5]. However, very few of them require nonsurgical management, and less than 1% require surgical procedures [6]. Dentists must be aware of the signs and symptoms of foreign body ingestion. In children, crowns, dislodged restorations, files during endodontic procedures, and extracted teeth are common objects for accidental ingestion [6-8]. It might require an extensive surgical intervention and occasionally leads to life-threatening situations if not appropriately managed. Therefore, dentists should be aware of the management and prevention of dental objects ingestion protocol. Hence, this case report describes a case of accidental stainless crown ingestion in a five-year-old boy who was managed per a management protocol.

## Case presentation

A five-year-old boy visited the pediatric dentistry clinic with pain in the upper left back tooth region. Based on clinical and radiographic examinations, he was diagnosed with a multi-surface caries lesion in the upper left first primary molar. It was decided to place a stainless steel crown, and the child was scheduled for the next appointment. Hall technique was used for crown placement, and the try-in was made. While performing the trial with the stainless steel crown for the fit, the boy suddenly moved, and due to excessive saliva in the mouth, the crown slipped out of hand. He closed his mouth and swallowed the stainless steel crown. He neither showed any signs nor discomfort. The operator attempted to retrieve the swollen crown by patting the boy on the back to spit the crown, and it was futile. Subsequently, he was taken to the emergency department in the Ministry of Health hospital to view abdominal and chest radiographs. The radiographic examination revealed the presence of a radiopaque foreign body in the stomach (Figure 1). The boy was asymptomatic, and the object ingested was observed to be small and blunt. Upon discussion with a physician, there were no risks for the boy, but it was decided to keep him under observation by the parents. The boy was advised to follow a fiber-rich diet to simplify the crown excretion. At 24 hours, the posteroanterior abdomen radiograph depicted the crown below the sacral level, very close to the anal region (Figure 2). The same afternoon, the crown was excreted with the patient's stool (Figure 3). 

**Figure 1:** Posteroanterior abdomen showing the stainless steel crown

**Figure 2:** Posteroanterior abdomen showing the presence of stainless steel crown at the sacral level

**Figure 3:** Stainless steel crown

The patient was scheduled for the next appointment to provide stainless steel crown.

## Discussion

Multiple authors have reported the ingestion of various foreign bodies, such as toy parts, coins, safety pins, magnets, and batteries. In a clinical dental setting, a patient's risk of aspirating a foreign body is increased by myriad factors, such as sedation, local anesthesia, supine and reclined positioning, jerky or unexpected movements, and excessive salivation. Foreign objects pass through the GIT in the majority of the cases and are excreted in days without any signs and symptoms or, in some cases, may cause peritonitis by lodging in the duodenum or colon [9,10]. Nevertheless, it is imperative to keep such pediatric patients under medical surveillance. The patient visited the emergency department and consulted a physician in the present case. The necessary radiographs were taken in 24 and 48 hours, which allowed to document the evidence of crown excretion through stool. In these cases, fiber-rich food is mandatory to excrete a foreign body through stools. A couple of authors suggested that bananas may be very beneficial in such instances [6-9]. In cases of foreign body ingestion, children may present with a variety of symptoms, including choking, drooling, and poor feeding in younger patients; dysphagia, odynophagia, and chest pain in older patients; or respiratory symptoms, especially in younger patients, due to tracheal compression or esophageal erosion [4,9,10]. A lateral cephalogram has been suggested if the child will become breathless or unable to explain the situation at the dental clinic [7,8,10].

Foley's catheter with endoscopy has been suggested to remove such foreign bodies; if it is not removed, open surgery or laparoscopy [5] has also been advocated in some cases. These management strategies are used only in cases with the signs mentioned earlier and symptoms. However, the patient showed neither any signs nor symptoms in the present case, and the ingested stainless steel crown was later excreted in the stool. Parental counseling also plays a significant role in such cases. Therefore, the boy's father was counseled by showing him previously published literature on the present case. Abdominal and chest radiographs have also been reported to essential in such cases. In the present case, the boy was planned to take abdominal and chest radiographs in 24-hours intervals, which could be advisable in non-symptomatic cases. Foreign body ingestion may cause damage to the airways or gastrointestinal mucosa, partial or complete airway obstruction, respiratory distress, post obstructive pneumonia, hemorrhage, or pneumothorax, intestinal perforations, or septic abscess [2-6]. It can be lethal if proper management is not taken. To avoid such instances in the dental operatory, use a rubber dam, attach dental floss to a stainless steel crown, place a gauge on the tongue, and slightly bend the child's head on the crown placement side. Over the decades, dentists have worked meticulously to prevent and minimize complications in the dental operatory through training. Hence, it is essential to have enough knowledge of the signs and symptoms of foreign body ingestion and aspiration.

## Conclusions

Accidental foreign body ingestion is not very uncommon in dental operatory among children. The awareness among the dentists regarding signs and symptoms of foreign body ingestion and aspiration is vital. Early diagnosis and proper management strategies with appropriate radiographs play a key role.
